The article "The Crucial Role of CXCL8 and Its Receptors in Colorectal Liver Metastasis" was retracted in 2023. Reasons: signs of a paper mill; suspected computer-generated content; unreliable results or conclusions; concerns about the data.

# The Crucial Role of CXCL8 and Its Receptors in Colorectal Liver Metastasis

**DOI:** 10.1155/2019/8023460

**Published:** 2019-11-20

**Authors:** Yaqin Bie, Wei Ge, Zhibin Yang, Xianshuo Cheng, Zefeng Zhao, Shengjie Li, Wenchao Wang, Yu Wang, Xiaofeng Zhao, Zhengfeng Yin, Yunfeng Li

**Affiliations:** ^1^Colorectal Surgery, Third Affiliated Hospital of Kunming Medical University, Tumor Hospital of Yunnan Province, Kunming, Yunnan 650118, China; ^2^Oncology, Taikang Tongji (Wuhan) Hospital, Wuhan, Hubei 430051, China; ^3^Molecular Oncology Laboratory, Eastern Hepatobiliary Surgery Hospital, Second Military Medical University, Shanghai 200438, China

## Abstract

CXCL8 (also known as IL-8) can produce different biological effects by binding to its receptors: CXCR1, CXCR2, and the Duffy antigen receptor for chemokines (DARC). CXCL8 and its receptors are associated with the development of various tumor types, especially colorectal cancer and its liver metastases. In addition to promoting angiogenesis, proliferation, invasion, migration, and the survival of colorectal cancer (CRC) cells, CXCL8 and its receptors have also been known to induce the epithelial-mesenchymal transition (EMT) of CRC cells, to help them to escape host immunosurveillance as well as to enhance resistance to anoikis, which promotes the formation of circulating tumor cells (CTCs) and their colonization of distant organs. In this paper, we will review the established roles of CXCL8 signaling in CRC and discuss the possible strategies of targeting CXCL8 signaling for overcoming CRC drug resistance and cancer progression, including direct targeting of CXCL8/CXCR1/2 or indirect targeting through the inhibition of CXCL8-CXCR1/2 signaling.

## 1. Introduction

CXCL8, also known as neutrophil-activating factor (NAF) and interleukin 8 (IL-8), was the first chemokine identified, and it was originally identified as a leukocyte chemoattractant [1]. CXCL8 is primarily produced by neutrophils, monocytes, macrophages, T cells, epithelial cells, and endothelial cells [2]. CXCR1, CXCR2, and DARC are three receptors for CXCL8 that produces different biological effects by binding to different receptors. The main effective receptors are CXCR1 and CXCR2, of which 80% have homologous sequences. CXCR1 and CXCR2 belong to the seven-transmembrane G protein-coupled receptor (GPCR) subfamily and are mainly expressed on leukocytes, endothelial cells, epithelial cells, and neuronal cells [2]. The atypical chemokine receptor DARC, however, is a seven-transmembrane protein that is not coupled to trimeric G proteins; it is expressed on neuronal cells, endothelial cells, and erythrocytes [3–5].

CXCL8 may control leukocyte trafficking during inflammation as well as during homeostasis, principally through interacting with the chemotaxis receptor CXCR1 [6], and it is necessary for the linkage between tumors and inflammation. CXCL8-mediated tumor progression, occurring primarily through CXCR1 and CXCR2, has been identified as a function of the modulation of angiogenesis, immune cell infiltration, cell motility, cell survival, and growth in the microenvironment as well as the regulation of local antitumor immune responses [7–9]. As an important CXC chemokine, CXCL8 was the first of the angiogenic chemokines that was found to contain the sequence Glu-Leu-Arg (the ELR motif), a potent inducer of angiogenic activity [10, 11]. The angiogenesis mediated by CXCL8 is sophisticated. If CXCL8 interacts with the receptor CXCR2, it plays a proangiogenic role, while the opposite role is played when interacting with the DARC receptor, which has been classified as a “silent” receptor that clears ELR^+^ angiogenic chemokines and inhibits tumor development [12, 13]. However, more researchers support that CXCL8 acts primarily as an angiogenic activator, which in turn establishes a venue for the local invasion, migration, and metastasis of cancer cells.

During the past decade, many studies have addressed the facilitation of CXCL8 in various types of cancer [14–20], among which colorectal cancer and its liver metastases are significantly associated with elevated CXCL8 signaling within the tumor microenvironment [16]. In addition to promoting angiogenesis, proliferation, invasion, migration, and survival of CRC cells, CXCL8 and its receptors have been known to induce the epithelial-mesenchymal transition (EMT) of CRC cells to help them to escape from host immunosurveillance and resist anoikis, which promotes the formation of circulating tumor cells (CTCs) and the colonization of distant organs (see Figure 1). Liver metastasis is the most important factor creating a poor prognosis in colorectal cancer, which is the main obstacle influencing the curative effects of the existent treatment. This review provides an overview of the established roles of CXCL8 signaling in CRC and subsequently discusses the possible strategies for targeting CXCL8 signaling in CRC drug resistance and progression, including indirect strategies (e.g., anti-inflammatory medications and NF-*κ*B inhibitors) and direct strategies, such as CXCL8 inhibition or inhibition of its receptors (e.g., neutralizing antibodies, small-molecule receptor antagonists, and siRNAs) (see Table 1).

## 2. CXCL8 and Its Receptors in the Promotion of the Invasion and Metastasis of CRC Cells and the Formation of CTCs

Considerable evidence has shown that EMT is a pathological process contributing to cancer invasion and metastasis. When EMT occurs in the epithelial tumor cells, they develop some characteristics of mesenchymal cells, such as reduced cell-cell adhesion, which can improve their invasive migration abilities and promote the movement of tumor cells from the extracellular matrix and their release into the blood or lymph. The tumor cells in the blood or lymph are called CTCs, and these become potential “seeds” for distant metastases.

### 2.1. Inducing EMT to Promote the Invasion and Metastasis of CRC Cells

Hwang et al. isolated colonospheres from 22 primary CRC tissues and several CRC cell lines and characterized their gene expression patterns by microarray analysis, including CXCL8, snail, and the colon cancer stem cell marker CD44, as well as the mesenchymal marker vimentin [21]. The results showed that snail could activate the expression of CXCL8 directly by binding to the E3/E4 E-boxes, a CXCL8 promoter region, and then regulate colon cancer stem cell activity and EMT in the cancer cells, which indicated that CXCL8 can interact with snail to induce EMT and promote the invasion and metastasis of CRC cells. In our published study, the results of immunofluorescence staining and Western blot showed that CXCL8 alone could induce increased expression of beta-catenin and the mesenchymal marker vimentin without being accompanied by changes in the expression of E-cadherin and cell morphology in CRC cells, which has been called “partial EMT” [22]. However, decreased expression of E-cadherin and increased expression of vimentin and/or beta-catenin, a total EMT-like phenotype in CRC cells, were obvious when another chemokine CCL20 was costimulated with CXCL8 (*P* < 0.01), and the process occurred along with the activation of the PI3K/Akt-ERK1/2 signaling pathway. After EMT, CRC cells can regulate CXCL8 in an autocrine manner and increase the expression of its CXCR1 and CXCR2 receptors, which could contribute to cancer progression, particularly to cancer invasion, dissemination, and metastasis. The antibody inhibition test showed that CXCR1 but not CXCR2 was active in this process [23]. In addition, Kobayashi et al. identified several genes with significantly different microarray signals between the tumor front and the tumor center [24]. Among these genes, six chemokines, including CXCL8, matrix metalloproteinase7 (MMP7), and EMT-related molecules, showed significant upregulation at the tumor front; nevertheless, the fold changes of MMP7 and EMT-related molecules were smaller than those of CXCL8, indicating that CXCL8 was more important than MMP7 and EMT-related molecules in the process of cancer cell invasion and metastasis distance. As EMT-associated proteins, CXCL8 [22] and MMPs [25] may cooperate with each other to induce EMT, invasion, and metastasis of CRC cells. Obviously, CXCL8 can participate in the process of EMT through a variety of means to promote CRC cell invasion and metastasis.

### 2.2. Promoting the Extravasation of CRC Cells and the Formation of CTCs

A variety of mesenchymal cells (such as neutrophils and endothelial cells) and blood flow shear stress are involved in the extravasation process of the tumor cells from the tumor tissue. In the adhesion assay of tumor cells to endothelial cells, Li et al. [26] found that when CXCL8 mRNA and protein expression in the CRC cells was higher, the CRC cells more strongly adhered to the endothelium (EC), and the permeability of the CRC cells was enhanced, proving the role of CXCL8 in the adhesion processes of colon cancer cells to endothelial cells. Additionally, in the parallel-plate flow assay, Liang et al. [27] discovered that tumor-liberated CXCL8, regulated by various shear stresses, could induce melanoma cell-PMN interactions mediated by the binding between intercellular adhesion molecule-1 (ICAM-1) on melanoma cells and *β*2 integrins on PMNs, which facilitate melanoma cell adhesion to the EC. After adhesion to the EC, the subsequent extravasation of the tumor cells by a shear rate-dependent mechanism was also regulated by endogenously secreted CXCL8 within the tumor microenvironment. This phenomenon indicated that CXCL8 can mediate the adhesion of tumor cells to the EC and the resulting exosmotic process into the peripheral blood. Identical results were found in similar tests of other types of tumor cells. Interestingly, cells grown at low density were more effective in invading endothelial monolayers than cells grown at high density. When maintained at low cell density, triple-negative human MDA-MB-231 breast cancer cells that were widely used for modeling cellular invasion showed an easily discernible endothelial monolayer invasive phenotype, which was associated with a YAP-dependent upregulation of the cytokines, including CXCL8. Antibody blockade of cytokine receptors (such as CXCR2) inhibited invasion and confirmed that they were rate-limiting drivers that promoted cancer cell vascular invasiveness [28]. This phenotypic discrepancy was also observed in a zebrafish model in which the cancer cells could travel into the vasculature after injection into the yolk sac and then extravasate into tissues from the vasculature. Therefore, after breaking away from the extracellular matrix, the tumor cells will be in a low-density state in which the CXCL8-CXCR2 signaling axis may promote tumor cell herniation through the blood vessels and then the release into the blood to form CTCs. The result that the expression of CXCL8 in cancer-adjacent tissue is higher than that in cancer center tissue seems to provide evidence to support this point of view [24].

## 3. CXCL8 and Its Receptors in the Survival Mechanisms of CRC Cells

Mechanistic analyses determine that CXCL8 and its receptors contribute to the survival of CRC cells, mainly by reducing the survival pressure of tumor cells and helping them become resistant to anoikis before and after invading the blood. Moreover, CXCL8 and its receptors are also involved in the mechanism of CRC cells and circulating CRC cells escaping from immune surveillance.

### 3.1. Contribution to the Survival and Resistance to Anoikis of CRC Cells and Circulating CRC Cells

Hypoxia [29], a representative feature of the tumor microenvironment, can stimulate the transcriptional activation of PPARơ (peroxisome proliferator-activated receptor ơ) through p300 and the PI3K/Akt pathway, leading to the expression of tumor-promoting cytokines, such as CXCL8 and VEGF (vascular endothelial growth factor) [30], which could promote the process of angiogenesis through acting on tumor cells as well as the EC. As a result, the neovascularization formed in the microenvironment would be able to provide adequate nutrition to sustain further growth and survival of tumor cells under a state of reduced oxygen pressure in tissues.

As is well known, the wild type of TP53 is an important broad-spectrum tumor suppressor molecule, but the mutated TP53 exhibits new oncogenic functions, such as the promotion of survival, proliferation, and invasion [31]. It has been reported that the CXCL8-TP53 signaling pathway plays a role in promoting tumor progression. For instance, the mutated TP53 in prostate neuroendocrine cells can inactivate the CXCL8-CXCR2-p53 pathway that universally inhibits cellular proliferation, leading to the development of small-cell neuroendocrine carcinoma (SCNC) [31]. Interestingly, in order to get a more comprehensive analysis of the CRC-related gene network, Sonachalam et al. [32] integrated previous knowledge from protein interactions and gene signatures with gene set enrichment analysis (GSEA) and protein/gene network modeling to identify the gene network signatures for CRC from gene expression microarray data; from this integration, several important subnetwork signatures for CRC were discovered, such as the TP53 subnetwork and the CXCL8 subnetwork, which correspond to apoptosis and the immune response, respectively. Therefore, the CXCL8-TP53 signaling pathway may play an important role in survival mechanisms of the CRC cells.

Autophagy, a catabolic process of cellular self-digestion that acts as a double-edged sword in tumor survival mechanisms and progression, is a potential target for antineoplastic therapies. On the one hand, the tumor cells can increase the level of autophagy themselves to relieve the survival pressure and resistance to apoptosis; on the other hand, excessive autophagy may be able to induce autophagic apoptosis, and the balance between proapoptotic and antiapoptotic effects directly affects the survival of the tumor cells. To obtain a more comprehensive understanding of the survival mechanisms of the tumor cells, it is very important to look for one or more specific markers reflecting the level of autophagy, which is difficult and costly to detect clinically. Kraya et al. [33] used ELISA to detect the levels of several major secretory proteins in melanoma cell culture medium before and after knocking out the autophagy-related gene; the researchers found that several biomarkers, including CXCL8, could become the candidate reflecting the level of autophagy in tumor cells to some extent. Moreover, to evaluate Toll-like receptor- (TLR-) mediated autophagy induction in intestinal epithelial cells (IEcs) and CRC cells as well as its relationship with proinflammatory productions of CXCL8, IEC-6, and HCT-15, cells were cultured with or without various TLR ligands, followed by evaluation of the expressions of CXCL8 by ELISA and real-time PCR. To reveal the status of autophagy in IEcs and CRC cells, light chain 3- (LC3-) II expression was examined using Western blotting and immunofluorescence with confocal microscopy. Additionally, the specific autophagy-related gene (Atg) 7 siRNA was transfected into IEcs, and the expression of CXCL8 was determined following exposure to various TLR ligands. As a result, the CRC cells treated with the TLR ligands could produce considerable amounts of CXCL8, but CXCL8 expression was downregulated, and after inhibiting Atg7, it was found that CXCL8 may be involved in survival mechanisms within the downstream signaling pathways of autophagy [34].

In our published study [35], we showed that CXCL8 expression was negatively associated with anoikis in CRC cells. We assessed the apoptosis of CRC cells under detachment and attachment conditions. As a result, there was no significant difference in the rate of apoptosis among the CRC cell lines when they were cultured under attachment conditions. Meanwhile, the suspension-cultured cells lost cell-cell adhesion, which resulted in a high apoptotic rate of CRC cells. These data indicated that CRC cells undergo apoptosis when cultured in suspension, similar to the majority of CTCs in the peripheral blood. We also showed that cell apoptosis stimulated by the loss of adhesion was inversely correlated with CXCL8 and TOPK expression. In addition, the CRC cells cultured under detachment conditions but not under attachment conditions enhanced their resistance to anoikis after CXCL8 treatment, which was coupled with the increase in TOPK and the activation of AKT and ERK. All of these findings indicated that a small number of circulating CRC cells would increase the expression of CXCL8 to resist anoikis in the bloodstream. However, the small amount of circulating cancer cells separated from the peripheral blood is currently difficult to use in subsequent experiments due to the immature technology relating to the culture and amplification of CTCs. How CXCL8 and its receptors regulate the survival and resistance to anoikis of CTCs has not yet been elucidated.

### 3.2. Helping CRC Cells and Circulating CRC Cells Escape from Immune Surveillance

Neutrophils are commonly known as “professional” phagocytic cells of the innate immune system, and CD56^+low^ NK cells are endowed with cytotoxic and cytokine-producing capacities. These two immune cells predominate in the peripheral blood, and more than 90% of them are equipped with CXCR1 and CXCR2 [36], which give them the ability to comigrate into sites of acute inflammation or tumors in response to their ligand CXCL8 as well as other ELR^+^ chemokines and to participate in the earliest phase of the innate immune response [37]. To study the role of the migration of CXCL8 into the tumor tissue of dendritic cells (DC), Alfaro and colleagues [38] developed mice whose peritoneums were injected with CRC cell lines, HT29 cells, CaCo2 cells, or SW480 cells, to induce subcutaneous tumors, and then, fluorescence-labeled DC was injected into the subcutaneous tissue 5 mm away from the tumor. As a result, fluorescence-labeled DC was attracted to the tumor tissue, and such migratory behavior was inhibited when DC was coinjected with a neutralizing anti-CXCL8 mAb. More importantly, preexposure of the DC cultures to CXCL8 for 24 h prior to injection also extremely impaired the migration towards the tumor tissue. Therefore, tumors can attract DC by means of CXCL8, but chronic exposure to CXCL8 desensitizes DC to this migration in vivo. Due to these effects, increased CXCL8 in the serum, the tumor microenvironment, and the adjacent tissues can impair the migratory orientation of DC to CRC tissue, which helps the CRC cells escape immune surveillance.

When tumor cells intrude into the blood, they are called CTCs. Despite the fact that most CTCs are killed by immune effector cells, a small number of them evade immune surveillance and survive in the blood, eventually resulting in clonal expansion and the formation of metastatic lesions. It is crucial to define the characteristics that enable a select CTC population to escape immune surveillance; in particular, it must be determined whether interactions between adhesive immune cells and CTCs provide a protective effect on CTC survival. To study human CXCL8, Asfaha and colleagues [39] developed a transgenic mouse that carried the entire human CXCL8 gene and associated regulatory elements encoded within a bacterial artificial chromosome. Using this model system, they showed that CXCL8 significantly accelerated inflammation-associated colonic carcinogenesis through increased recruitment of myeloid-derived suppressor cells (MDSCs), a large population of immature myeloid cells. MDSCs can induce strong systemic and local immunosuppression, a phenomenon that has been proven to facilitate cancer invasion and distant metastasis. Therefore, Liu et al. [40] hypothesized that CTCs can create a defensive shield consisting of adhesive MDSCs that allow the evasion of immune surveillance. A variety of cytokines, including CXCL8 secreted by MDSCs, were pivotal for promoting the growth and proliferation of CTCs in the shield. However, this phenomenon has been reported in CRC. Katoh et al. [41] presented genetic evidence showing that the loss of CXCR2 dramatically suppressed colitis-associated tumorigenesis by inhibiting the infiltration of MDSCs into the colonic mucosa and tumors in a mouse model of colitis-associated CRC induced by feeding AOM/DSS. As the ligand of CXCR2, levels of CXCL8 were elevated in the inflamed colonic mucosa and CRC tissue and induced MDSC chemotaxis via CXCR2. Then, MDSCs accelerated tumor growth through inhibiting CD8^+^ T cell cytotoxic activity, which damaged the immune response. Therefore, CXCL8 and its receptors may act as a defensive shield for escaping immune surveillance of the tumor cells as well as CTCs. Above all, the finding that CXCL8 levels towards the center of cancer tissue are lower than those towards cancer-adjacent tissue [24] seems to provide evidence of this view.

Furthermore, to evaluate the influence of the innate immune response marker TLR ligands on autophagy-mediated innate immune responses, Li et al. [34] transfected Atg7-specific siRNA into IEcs and determined the CXCL8 expression of the CRC cell HCT15 after exposure to various TLR ligands. The results showed that Atg7 gene expression silencing led to downregulation of TLR-mediated CXCL8 expression in IEcs and CRC cells, which indicated a potential role of autophagy in generating innate immune responses. As the upstream signaling pathways of CXCL8, autophagy may be an important intracellular mechanism to induce the innate immune system through upregulating the expression of CXCL8 by TLRs [34].

## 4. CXCL8 and Its Receptors in the Chemotaxis of Circulating Tumor Cells to the Liver

Over the years, the “seed and soil” doctrine and the theory of the inflammatory microenvironment have received more and more attention. That tumor cells are able to transfer to a specific organ and then grow there is mainly related to the suitable “soil” provided for the tumor cells in the target organ. The inflammatory microenvironment is also active in the tumor development and transfer processes. In the breast cancer lung metastasis model of mice, Wculek and Malanchi [42] found that before breast cancer cells infiltrated the premetastatic lung tissue, CD11b^+^Ly6G^+^ neutrophils, the mainly excretive cells of CXCL8, accumulated in the lung first and then facilitated the metastatic cancer cell transfer to the lung. As an important neutrophil chemotactic factor, CXCL8 is likely to play a significant role in the aggregation of neutrophils to the metastases, and in return, the aggregate neutrophils will secrete more CXCL8. This cascade effect contributes to the formation of the premetastasis inflammatory microenvironment and the preparation for the homing of tumor cells (i.e., nesting first and then homing). Therefore, we have reason to speculate that CXCL8 aggregated in the premetastases would be the key chemotactic factor in the homing of CTCs. Moreover, to identify candidate tumor-derived attractants for CTCs, Kim et al. [43] compared the secreted levels of 180 cytokines in conditioned media and found that the levels of several cytokines were higher, including CXCL6, CXCL8, oncostatin M, and vascular endothelial growth factor, among which CXCL6 and CXCL8 showed the sharpest increases. Next, they developed a CTC model by injecting the tumor cells into the tail vein of mice to study the role of CXCL8 in tumor self-seeding of CTCs. As a result, they found that the tumor-derived cytokine CXCL8 acted as a CTC attractant that could induce the migration and colonization of CXCR1/2^+^ tumor cells to CXCL8 high expression sites. This phenomenon disappeared when the tumor cell CXCR1/2 was knocked out, indicating that CXCL8 may attract CXCR1/2^+^ CTCs homing to the primary tumor or metastases. In another study, Li et al. [26] observed a differential expression of CXCL8 and its receptors, CXCR1 and CXCR2, in human CRC cells with different metastatic potentials by adding a certain amount of exogenous CXCL8 to their culture medium; in this study, the mRNA and protein expression levels of CXCL8 as well as CXCR1 and CXCR2 were significantly lower in nonmetastatic (Caco2 cells) and low metastatic (KM12C cells) CRC cells than in high metastatic (KM12L4 cells) CRC cells. Additionally, antibody inhibition experiments supported a key role of CXCR1/2 in the migration process of CRC cells, which suggested that CXCL8 and its receptors improved the metastatic potential along with the migration ability of CRC cells. These results indicated a domino effect of CXCL8 and its receptors on the homing process of CTCs; when CXCR1/2 expression on CTCs is higher, the metastasis occurring under the chemotactic role of CXCL8 is easier.

## 5. CXCL8 and Its Receptors in the Process of MET and Colonization of Circulating CRC Cells

Mesenchymal-epithelial transition (MET), as the inverse process of EMT, reverses tumor cells that have undergone EMT to an epithelial cell state, making them easy to integrate into new tissues and organs and form metastases. In our recent study mentioned above [22], we showed that CXCL8 alone could only induce pEMT in CRC cells, and this semiconservative epithelial characteristic provides a significant contribution to the subsequent recovery of epithelial characteristics, namely, MET. In general, the dynamic transformation between the epithelial phenotype and mesenchymal phenotype of tumor cells is regulated by CXCL8 in the tumor microenvironment.

Osteopontin (OPN) is widely distributed in various tissues and cells and is involved in tissue repair, self-metabolism, and other functions that allow OPN to play an important role in tumor metastasis [44–46]. Presently, it has been shown that OPN is related to both the EMT and MET processes of tumor cells. In previous studies, Dong et al. [47] indicated that OPN can induce EMT of HCC cells by increasing vimentin stability, which provided a more in-depth understanding of the molecular mechanisms of OPN in promoting HCC metastasis and opened tantalizing therapeutic possibilities in HCC. To gain more insights into the interaction between OPN and vimentin, the regions of vimentin responsible for their binding were mapped, and the results indicated that OPN only bound vimentin deletion mutants, including the central rod domain and deletion of the rod domain was adequate to abolish binding of vimentin to OPN. Liang [48] transfected lentivirus into tumor cells to upregulate/downregulate OPN expression and found that the nuclear expression of OPN increased cadherin expression, induced MET of tumor cells, and remodeled the epithelial phenotype of tumor cells, which suggested that the dynamic transformation process of the epithelial phenotype-mesenchymal phenotype-epithelial phenotype in tumor cells was inseparable from the role of OPN. It is worth noting that there is a complicated relationship between CXCL8 and OPN. Functional genomic analysis showed that the engagement of the integrin receptors avb3 and a5b1 of OPN and FN, respectively, had significant effects on chondrocyte functions. Ligation of avb3 and a5b1 using activating mAb JBS5 and LM609 (which act as agonists similar to OPN and FN N-terminal fragments) regulated the CXCL8 cytokines as well as the inflammatory mediators such as NO and PGE2. These data demonstrated a cross talk in signaling mechanisms between OPN and CXCL8 inflammatory cytokines [49].

It has been demonstrated that OPN has chemotactic activity for leukocytes, which is involved together with CXCL8 in prostate cancer recurrence [50]. What is more, OPN contributes to the remodeling of the extracellular matrix (ECM) and to the development of angiogenesis, a function also shared by CXCL8 [51]. To study the relationship between OPN and CXCL8, Erreni et al. [52] investigated the expression of OPN and CXCL8 in CRC samples by using qRT-PCR. As a result, there was a significant increase in both mRNA OPN and CXCL8 in tumor tissues compared to the normal mucosa (*P* < 0.0001), and they found a prominent linear correlation between OPN and CXCL8 mRNA expressions in tumor tissues, indicating that there was a synergistic role between CXCL8 and OPN in regulating the development of colorectal cancer. Overall, they can not only coregulate the motility, chemotaxis, and shaping of cancer cells but also synergistically induce the MET process of CRC cells.

PMNs in the peripheral blood can not only promote tumor cell adhesion to the endothelial cell and extravasation into the blood but also participate in the adhesion and colonization of the target organ by CTCs via CXCL8 and the ICAM-1-*β*2 integrin signaling pathway [27]. Using in vivo models of metastasis, Spicer et al. [53] found that neutrophils facilitated the adhesion of cancer cells and CTCs within liver sinusoids and thereby influenced metastasis in the CXCL8-ICAM-1-*β*2 integrin signaling pathway. Intravital microscopy demonstrated that cancer cells could adhere directly on top of the arrested neutrophils, indicating that neutrophils may act as a bridge to promote interactions between cancer cells and the liver parenchyma.

## 6. CXCL8 and Its Receptors in the Growth and Progression of CRC and Its Liver Metastases

CXCL8 and its receptors are involved not only in mediating interactions between tumor cells and stromal cells but also in regulating the tumor microenvironment in primary CRC as well as its liver metastasis and promoting colorectal cancer progression by inducing angiogenesis, regulating tumor-associated stroma, or acting directly on tumor cells. Numerous clinical studies, including our research, have demonstrated that the elevated levels of CXCL8 in serum and tissues from colorectal cancer patients were related to the grade, stage, lymph node metastasis, and liver metastasis of CRC (*P* < 0.05), while the survival curve analysis also showed that the significantly decreased disease-free survival (DFS) and overall survival (OS) (*P* < 0.05) were highly related to the high expression of CXCL8 in CRC patients, which led to tumor progression and a poor prognosis [22, 35, 54, 55].

### 6.1. Indirect Effect on Promoting the Growth and Proliferation of CRC Cells

Recently, mesenchymal stem cells (MSCs) have been shown to home to carcinoma and facilitate the formation of the tumor-associated stroma. Wang et al. [56] reported that CXCL8 was the highest upregulated proangiogenic factor in MSCs that were cocultured with CRC cells, and it was expressed at substantially higher levels in MSCs than in CRC cells. To evaluate the effect of mesenchymal stem cell- (MSC-) derived CXCL8 on CRC angiogenesis and growth, they used MSCs that expressed interfering (small hairpin) RNAs (shRNA) targeting CXCL8 (shCXCL8-MSCs). They found that MSC-secreted CXCL8 promoted the proliferation, migration, and tube formation ability of human umbilical vein endothelial cells (HUVEC), which revealed the fact that CXCL8 induced angiogenesis in the tumor microenvironment to indirectly promote the growth and proliferation of cancer cells. Additionally, this phenomenon was also observed in in vivo studies. Apart from MSCs, tumor-associated fibroblasts, pericytes, and endothelial cells are also stromal cells in the tumor microenvironment. Ijichi et al. [57] showed that several CXC chemokines secreted by the pancreatic ductal adenocarcinoma (PDAC) cells in K-ras^+^Tgfbr2^KO^ mice induced connective tissue growth factor (Ctgf) expression in tumor-associated fibroblasts, which enhanced the growth of PDAC cell allografts but not the PDAC cells themselves; the tumor progression was attenuated by CXCR2 inhibition, which indicated that tumor-stromal interactions regulated tumor progression via a CXCR2-dependent chemokine and Ctgf axis. Singh et al. [58] found that the proliferation and migration ability of endothelial cells would be significantly inhibited when the expression of CXCR1/2 in endothelial cells was knocked out, suggesting that CXCL8, the ligand of CXCR1/2, may contribute to angiogenesis and provide adequate nourishment to the cancer cells, resulting in tumor progression. In addition, to study the role of CXCL8-CXCR1/2 in the growth of colorectal liver metastasis, Varney et al. [59] established mice whose spleens were injected with KM12L4 tumor cells to induce colorectal cancer, and a CXCR1/2 antagonist was used to interrupt the CXCL8-CXCR1/2 signal. After three weeks, they resected the primary splenic tumors and liver metastases, portions of which were processed for immunohistochemistry, and the remaining portions were lysed for protein and RNA studies. As a result, the microvessel density of the liver metastases from the mice treated with a CXCR1/2 antagonist was lower than that from the control group. All these findings indicate that CXCL8 and its receptors can act on the tumor-associated stromal cells to indirectly regulate the growth and proliferation of CRC cells by promoting angiogenesis and regulating the tumor-associated stromal environment in the primary tumor as well as the metastases.

### 6.2. Direct Effects on Tumor Cells to Promote the Growth and Proliferation of CRC Cells

CXCL8 and its receptors can affect the tumor cells directly to promote their growth and proliferation. Lee et al. [16] developed an immunodeficient and skin-specific CXCL8-expressing transgenic model to evaluate colorectal cancer growth as well as metastasis and grafted syngeneic mouse colorectal cancer cells in CXCR2-knockout (KO) mice to study the contribution of CXCR2 to cancer progression in the microenvironment. The results showed that increased expression of CXCL8 in the tumor microenvironment and serum profoundly enhanced the growth of human and mouse colorectal cancer cells with increased peritumoral angiogenesis, and it also facilitated the extravasation of the cancer cells into the liver. Moreover, the tumor growth was inhibited in CXCR2-KO mice with increased tumor necrosis and reduced tumor angiogenesis, which indicated that the elevated levels of CXCL8 in the tumor microenvironment enhanced colorectal cancer growth and the absence of CXCR2 prevented the growth. Also in the CXCL8 transgenic model, Asfaha et al. [39] found that the high CXCL8-expressing transgenic mice were more likely to develop colorectal tumors when fed azoxymethane and polyglucosan sodium sulfate, and the most import factors in promoting the tumor progression were the immature myeloid cells accumulated in the tumor microenvironment as well as the CXCL8 secreted by these immature myeloid cells. Wu et al. [60] found that the CXCL8 in CRC tissues played a role in the leukemia inhibitory factor receptor- (LIFR-) induced angiogenesis; the depletion of CXCL8 brought about a decreased angiogenic activity of LIFR in CRC cells.

Furthermore, CXCL8 is highly expressed not only in primary tumors but also in the metastases. Compared with the corresponding neighboring tissues, Rubie et al. [61] showed that CXCL8 protein and mRNA expressions were significantly upregulated in all pathological tumor tissues, including the primary CRC tissues as well as the colorectal liver metastasis (CRLM). However, the upregulation amplitude in synchronous or metachronous CRLM was much stronger than that in the corresponding primary CRC tissues (*P* < 0.05), and CXCL8 expression was significantly higher in CRLM than in primary CRC tissues. This concentration gradient of CXCL8 would be a pivotal factor inducing CRC cells to metastasize to the liver in a chemotactic pathway. Moreover, when the metastases form, more and more CXCL8 will be secreted in the tumor microenvironment to accommodate the growth of metastases, and the role of CXCL8 seems to be more important in metastasis than in primary CRC tissues. In the CRLM model, not only did Varney et al. [59] find that the microvessel density in liver metastases from mice treated with a CXCR1/2 antagonist is lower but they found that the apoptosis rate of the tumor cells was also higher in the CXCR1/2 antagonist-treated groups than in the control groups, which indicated that the CXCL8-CXCR1/2 signal axis promoted the growth and survival of tumor cells in the liver metastases.

## 7. Targeting CXCL8 and Its Receptors in CRC Progression and Drug Resistance

Surgical resection is the primary therapeutic approach for CRC, but distant metastasis or recurrence is the main reason influencing the curative effect of the radical surgery, which indicates a poor prognosis of malignant tumors. Therefore, it is particularly significant for patients being treated with drugs to improve the curative ratio before and/or after the surgery. However, drug resistance to conventional antineoplastic therapies is a serious issue. CXCL8 and its receptors are involved in almost the entire process of colorectal cancer progression. Targeting CXCL8-CXCR1/2 signaling axes may be a potential new therapeutic strategy to control CRC progression and overcome the drug resistance of colorectal cancer.

### 7.1. Targeting CXCL8 and Its Receptors in CRC Progression

The possible strategies of targeting CXCL8-CXCR1/2 signaling in CRC include indirect strategies (e.g., NF-*κ*B inhibitors and anti-inflammatory medications) and direct CXCL8 or CXCR1/2 blocking (e.g., neutralizing antibodies, small-molecule receptor antagonists, and siRNA strategies).

#### 7.1.1. Indirect Targeting

CXCL8-CXCR1/2 signaling may be targeted not only directly by regulation of CXCL8/CXCR1/CXCR2 expression and signaling but also indirectly by the regulation of significant signaling pathways and transcription factors, including PI3K/Akt, MEK/ERK, and NF-*κ*B, which are responsible for the regulation of CXCL8 and CXCR1/CXCR2 expression. It has been reported that CXCL8 was downregulated in the HT-29 CRC cell line after treatment with the PI3K/Akt inhibitor LY294002 [62]. Furthermore, neurotensin- (NT-) induced CXCL8 mRNA expression and protein secretion was inhibited when treated with both U0126 and PD98059, which blocked ERK activation in HCT116 cells [63], indicating that the MEK/ERK pathway was involved in CXCL8 regulation by NT. Interestingly, neither U0126 nor PD98059 completely blocked NT-induced CXCL8 mRNA, which showed both ERK-dependent and ERK-independent (such as NF-*κ*B) regulation of the CXCL8 gene by NT in HCT116 cells. What is more, curcumin, which blocked NT-mediated NF-*κ*B induction, and BAPTA-AM, a Ca^2+^ chelator, both inhibited CXCL8 mRNA expression and protein secretion in HCT116 cells. The inhibition of CXCL8 was then found to inhibit the growth and migration of HCT116 cells [64]. Strategies to target these signaling pathways and transcription factors may therefore attenuate CXCL8 signaling in CRC cells indirectly.

In addition, to determine the association with colorectal cancer risk and overall survival, Bondurant et al. [65] detected genetic variations in genes from various anti-inflammatory and proinflammatory interleukins, finding that CXCL8, CXCR1, and CXCR2 were all significantly associated with the risk and poor prognosis of colorectal cancer, which was significantly associated with the use of nonsteroidal anti-inflammatory drugs (NSAIDs), such as aspirin and ibuprofen. A landmark study in 1997 showed that low-dose aspirin was able to drastically reduce the risk of developing colon cancer [66], and subsequent randomized trials also demonstrated that the use of NSAIDs was correlated with a reduced risk of developing colon cancers [67]. Phosphorylated ibuprofen can also prevent the development of colorectal cancer by inhibiting NF-*κ*B activity [68]. Although the precise mechanisms by which NSAIDs prevent tumor development remain unclear, it is likely to be through COX-independent and COX-dependent mechanisms. Existing evidence highlights the importance of the inflammatory microenvironment in the growth and survival of tumor cells; therefore, the use of NSAIDs that reduce CXCL8 expression would play an important role in developing therapeutic strategies for CRC.

#### 7.1.2. Direct Targeting

As previously mentioned, CXCL8-induced migration of endothelial cells and the growth, proliferation, and migration of tumor cells as well as the chemotaxis of CTCs to the metastases can all be abrogated by neutralizing antibodies of CXCL8/CXCR1/CXCR2 or small-molecule receptor antagonists of CXCR1/CXCR2, indicating that directly targeting CXCL8-CXCR1/2 signaling is critical to controlling the CXCL8-mediated CRC progression. To study the role of small-molecule receptor antagonists in tumor progression, Varney et al. [59] established a mouse model of colorectal metastatic tumors and found that treatment with small-molecule antagonists of CXCL8 receptors resulted in the reduced survival of tumor cells and inhibited the tumor microenvironment as well as angiogenesis in mice, which controlled the tumor development and increased the survival of the mice. Gelfo et al. [69] highlighted the collective contributions of the inflammatory cytokine CXCL8 to the reduced sensitivity to EGFR blockade and suggested that inhibition of CXCL8 in combination with cetuximab may yield an effective treatment strategy for CRC patients refractory to anti-EGFR targeting. According to the expression levels of CXCL8 and/or its receptors in the serum, tumor tissue, and CTCs, as well as other clinical parameters, we may develop monotherapy or even combination therapies based on therapeutic strategies targeting CXCL8-CXCR1/2 signaling and other therapies such as immunotherapy to achieve successful treatment. Generally, monotherapy is less effective than combination therapy, which can inhibit tumor development from several aspects simultaneously and reduce the occurrence of drug resistance.

Immunotherapy has recently become a hot topic in the field of cancer therapy. CXCL8 and its receptors can induce the recruitment of tumor-associated immune cells into the tumor sites, which inhibited the activity of CD8^+^ T cells and thus helped the tumor cells to escape from immune surveillance [38]. Otherwise, PD1 signaling on T cells is one of the most important mechanisms for tumor cells escaping from host immune responses, but interruption of this axis alone only induces meaningful antitumor effects in a minority of cases, suggesting that other mechanisms are also involved in contributing to the immune evasion. To study the detailed mechanisms affecting this immunotherapy, Highfill et al. [70] developed a model of rhabdomyosarcoma in mice and found that the accumulation of CXCR2^+^CD11b^+^Ly6G^hi^ MDSCs in the tumor bed was the root cause limiting the efficacy of PD1 checkpoint blockade in cancer. MDSC^CXCR2+^-mediated suppression of antitumor immunity was just a local phenomenon because inhibition of MDSC^CXCR2+^ trafficking to the tumor enhanced the potency of PD1 checkpoint blockade, which indicated that combining CXCR2 inhibitors with immune checkpoint inhibitors may become a new combination immunotherapy strategy in cancer.

In addition, because the autophagy-CXCL8 signaling axis is one of the potential mechanisms in cellular resistance to apoptosis, targeting both autophagy and CXCL8 may provide double antitumor effects. Since autophagy plays a dual role in the development of colorectal cancer, we should determine what role autophagy plays in each patient first and then establish a combination therapy, including CXCL8/CXCR1/CXCR2 antagonists and autophagy inhibitors/activators, to enhance the antitumor effects according to the CXCL8/CXCR1/CXCR2 and autophagy expression levels of the patient. These combination therapies based on CXCL8 and its related signaling would provide a new breakthrough in tumor therapy.

### 7.2. Targeting CXCL8 and Its Receptors in CRC Drug Resistance

Primary or acquired resistance to conventional chemotherapeutic drugs is a general phenomenon that causes failure to antitumor therapy. Many molecular mechanisms have been found to be involved in drug resistance: apoptotic resistance or activation of survival signaling pathways, DNA damage repair, mutation of drug targets, alterations in drug metabolism, and increased rates of drug efflux, in which apoptotic resistance of cancer cells during treatment with conventional therapeutic drugs is the fundamental mechanism of drug resistance in antitumor therapy. As CXCL8 and its receptors play an important antiapoptotic role in the survival of CRC cells, targeting CXCL8 and its receptors could become a new strategy to reverse drug resistance in CRC therapy.

Hypoxia in the tumor microenvironment can induce the expression of CXCL8 and CXCR1/2, which allows the hypoxic cancer cells to be able to tolerate etoposide, a chemotherapeutic drug that works via DNA damage. When CXCL8 expression was inhibited, the efficacy of etoposide was significantly enhanced, suggesting that CXCL8 contributed to the apoptotic resistance and subsequent drug resistance [71]. Dabkeviciene et al. [72] determined the transcription levels of CXCL8, CXCR1, and CXCR2 in HCT116 and HCT116/FU cells, which was a subline derived from HCT116 cells resistant to 5-fluorouracil through a prolonged incubation with 5-FU, and found that the expression of CXCL8 and CXCR2, but not CXCR1, in HCT116 cells was significantly higher than that in HCT116/FU cells. Furthermore, after treatment with 5-FU, the expression levels of CXCL8 mRNA in HCT116 and HCT116/FU cells were 3.7- and 4-fold higher, respectively, than those in untreated cells, indicating that CXCL8 was upregulated in the chemoresistant subline of the CRC cell line HCT116, and modulation of the CXCR2 pathway was able to become a target for proliferation inhibition of chemoresistant CRC cells. Additionally, Ning et al. [15] inhibited the overexpression of CXCL8 in CRC cells by using small interfering RNA and found that the phenomenon of cancer cells resistant to oxaliplatin was significantly reduced, suggesting that the overexpression of CXCL8 in the cancer cells caused obvious resistance to oxaliplatin. This resistance to oxaliplatin was subsequently reversed under the combination of CXCL8/CXCR1/CXCR2 antagonists or neutralizing antibodies with oxaliplatin, which greatly improved the efficacy of oxaliplatin.

Above all, the upregulation of CXCL8 and its receptors is an obstacle to improving the efficacy of conventional chemotherapeutic drugs [69], and the combination with antagonists or neutralizing antibodies of CXCL8/CXCR1/CXCR2 may be a new strategy to reduce drug consumption, improve efficacy, and even reverse the drug resistance of clinical drugs, such as oxaliplatin, 5-FU, and capecitabine.

## 8. A Potential New Biomarker or Imaging Technology on CRC

Most intestinal diseases, including colorectal cancer, need endoscopy to make a clear diagnosis. However, for some chronic and recurrent intestinal diseases, frequent endoscopy also has a certain risk. Many patients refuse the endoscopy because of the creativity. Therefore, the emergence of a new biomarker or imaging technology is particularly important. In order to detect and locate the disease activity of patients with IBD with (99 m) tc-cxcl8 SPECT, Aarntzen et al. [73] injected 400 MBq Tc-99m CXCL8 to 30 patients of IBD separately and then performed their imaging, which included the planar after 30 min of the injection and SPECT acquisitions of the abdomen after 4 h of the injection. Results showed that the overall sensitivity and specificity for the detection was 71% and 70% for endoscopy and 95% and 44% for Tc-99m-CXCL8 scan. As the same as IBD, CXCL8 is also largely accumulated in the tumor microenvironment of CRC [74]. Consequently, the Tc-99m-CXCL8 scintigraphy may be a novel biomarker or imaging technique on the intestinal diseases.

## 9. Conclusion

Although CXCL8 and its receptors play a variety of roles in the process of colorectal liver metastases, the explicit mechanism of CXCL8 and its receptors in the resistance to anoikis and the immune tolerance of circulating cancer cells as well as the chemotaxis for CTCs homing to the liver remain unclear. Currently, the importance of accurate medical therapy is widely recognized in the field of cancer therapy, and monotherapy and combination therapies based on therapeutic strategies targeting CXCL8-CXCR1/2 signaling and other therapies could become an important route for preventing cancer recurrence and distant metastases. Because neutralizing antibodies and small-molecule antagonists of CXCL8 and its receptors have been used in various preclinical trials including colorectal cancer, they will be applied in clinical practice in the near future if the efficacy and specific treatment standards are sufficiently verified in clinical trials.

## Figures and Tables

**Figure 1:** CXCL8 and its receptors (CXCL8-R) are involved in almost the entire process of colorectal cancer progression and metastasis. First, CXCL8 and CXCL8-R promote CRC cell proliferation, invasion, migration, and angiogenesis and induce the epithelial-mesenchymal transition (EMT) of CRC cells, which contributes to the adhesion and intravasation of CRC cells to the blood. When tumor cells intrude into the blood, they are called CTCs, and most are killed by immune effector cells. However, a small number of them can evade immune surveillance and survive in the blood, which cannot be separated from the role of CXCL8 in inducing the anoikis resistance of CTCs, immune resistance, and autophagy. As a result of blood flow and the chemotaxis of the CXCL8 axis, CTCs may travel long distances, especially to the liver. After extravasation from the blood, the CRC cells induce the mesenchymal-epithelial transition (MET) and then colonize to form metastatic lesions. Targeting the CXCL8/CXCL8-R signaling axes may be a potential new therapeutic strategy to control cancer progression of and overcome drug resistance in colorectal cancer.

**Table 1:** A summary of potential new therapeutic strategies by targeting CXCL8-CXCR1/2 signaling axes alone or in combination with other treatments to control CRC progression and overcome drug resistance in colorectal cancer.

Targeting CXCL8-CXCR1/2 signaling axes alone		Combined with other treatments
Indirect targeting	Direct targeting	
NSAIDs (e.g., aspirin and ibuprofen)	CXCL8/CXCR1/CXCR2 siRNA, antagonist-neutralizing antibodies, small-molecule receptor antagonists (e.g., SCH-527123 and SCH-479833)	+Immunotherapy (e.g., PD1 checkpoint blockade)
PI3K/Akt inhibitor LY294002; a Ca^2+^ chelator, BAPTA-AM; ERK inhibitors U0126 and PD98059; NF-*κ*B inhibitor		+Conventional chemotherapeutic drugs (e.g., capecitabine, oxaliplatin, and 5-FU)
		+Autophagy inhibitors/activators
